# An Exploratory Cohort Study of the Association between the Level of Testosterone and Suicidal Ideation in Hospitalized Adolescent Females with Depression in China

**DOI:** 10.1155/2021/3529147

**Published:** 2021-10-27

**Authors:** Yan Liu, Shaohua Wang, Chuang Xue, Xiwen Hu, Guoling Zhou, Yuanyue Zhou, Dan Fang, Kaijing Ding

**Affiliations:** ^1^Department of Child and Adolescent Psychiatry, Affiliated Mental Health Center & Hangzhou Seventh People's Hospital, Zhejiang University School of Medicine, Hangzhou 310007, China; ^2^Division of Psychological Evaluation, Affiliated Mental Health Center & Hangzhou Seventh People's Hospital, Zhejiang University School of Medicine, Hangzhou 310007, China; ^3^Division of Depressive Disorder, Affiliated Mental Health Center & Hangzhou Seventh People's Hospital, Zhejiang University School of Medicine, Hangzhou 310007, China; ^4^Department of Clinical Laboratory, Affiliated Mental Health Center & Hangzhou Seventh People's Hospital, Zhejiang University School of Medicine, Hangzhou 310007, China

## Abstract

**Background:**

To date, around 4 per 100,000 adolescents committed suicide within the 29 OECD countries. The suicidal behavior is related to psychological factors, genetics, neurobiology, and other biomarkers. The aim of this study was to examine risk factors for the development of suicidal ideation in adolescent females with depression, focusing on the relationship between different testosterone levels and suicidal ideation, in order to help develop strategies to intervene in suicidal behavior in female adolescents with depression.

**Method:**

In this single-center prospective cohort study, we enrolled adolescent females with depression. We collected information on their baseline data, testosterone levels, symptom self-rating scale scores, suicidal ideation, non-suicidal self-injurious (NSSI) behaviours, and suicide attempts. We used multivariate logistic regression to identify risk factors for the development of suicidal ideation in adolescent females with depression.

**Results:**

A total of 113 hospitalized adolescent females were enrolled with a mean age of 13.5 (1.20). Among these patients, there were 86 (76.11%) subjects who suffered from suicidal ideation, 59 (52.21%) had NSSI and 23 (20.35%) had suicide attempt behavior. In the final model, higher level of testosterone (*p*=0.04) and higher age (*p*=0.02) were associated with the higher odds of having suicidal ideation.

**Conclusion:**

In this exploratory cohort study, the emergence of suicidal ideation was common among adolescent females with depression. This study is consistent with the other studies. It shows that the age is a potential predictor for suicidal ideation in hospitalized adolescent females with depression.

## 1. Background

The adolescent suicide problem is becoming a public health issue in recent years. According to the survey among 10–19-year-old adolescents from 29 OECD countries, the average suicide rate is 3.9 (1.80) per 100,000 people [1]. In childhood, the prevalence of mood disorders is relatively low (<1%), and the prevalence of mood disorders is similar in boys and girls, and sometimes the incidence in boys is even slightly higher than that in girls. However, the incidence of mood disorders in adolescents rises considerably after adolescence, up to 14%, with the incidence of mood disorders in females gradually increasing and surpassing that of males, with a male to female ratio of approximately 1 : 2 [2–4]. The reasons for the spike in prevalence during adolescence may be related to the physiological, hormonal, and psychological changes that occur during adolescence as well as changes in social roles [5].

Unlike adult depression, adolescent depression is characterized by extreme irritability, rather than low mood or anhedonia [6]. In addition, compared with adult depression, adolescent patients are more likely to experience extreme irritability, self-harm, and impulsive suicidal behaviors [7]. During the adolescence, compared with males, females are more prone to self-harm and suicidal behavior; especially between the ages of 12 and 15, the ratio of males to females reaches 1 : 5-6. However, as the age increases, the incidence of self-harm between male and female tends to be equal [8, 9]. Adolescent depression can seriously affect patients' academic performance and occupational capability [10, 11] and increase the risk of smoking and drug abuse [12]. Although most adolescents can recover from the initial depressive episode, 50%–70% will relapse within 5 years [13, 14]. Furthermore, depression in adolescence is related to anxiety, drug abuse, suicidal behavior, and unemployment in the adulthood [15, 16].

Adolescence is a period characterized by rapid changes in the brain, during which excitatory synapses are reduced, and the myelin sheaths in the frontal, temporal, and parietal regions increase to promote mood regulation, impulse control, and executive functions, which are more likely to lead to the occurrence of high-risk impulsive behaviors such as self-harm and suicide [17–19]. In contrast, testosterone levels will increase significantly during puberty compared to prepubescence, which can have a direct impact on the function of the central nervous system in adolescents [20].

Testosterone is a steroid hormone secreted by the testes in men or by the ovaries in women and to a lesser extent by the adrenal glands. In addition to its androgenic effects, which promote and maintain male secondary sexual characteristics, testosterone also promotes protein synthesis and stimulates the growth of bones, skeletal muscles, hair, and skin. It has been shown that testosterone levels change dramatically during adolescence and are strongly associated with mood disorders, self-harm, and suicidal behavior in adolescents [21]. Testosterone can cross the blood-brain barrier and affect the brain; testosterone can regulate many neurotransmitters or their receptors, including GABA, dopamine and serotonin (5-HT), etc., thereby affecting mood and behavior [22]. Previously, it seems that high testosterone levels and low levels of testosterone are both associated with the suicidal behavior [23–28]. There is argument that the age is the factor for the difference [25]. However, the gender difference and the association between adolescent female patients with depression and the level of testosterone are not clear.

## 2. Method

### 2.1. Study Design

This study is a convenience sampling, single-center, cohort study. The adolescent female subjects between the ages of 10 and 16 who were diagnosed with depressive disorder according to the International Classification of Diseases 10 (ICD-10) were eligible for this study.

### 2.2. Study Setting

The Seventh People's Hospital of Hangzhou (Mental Health Center of Zhejiang University School of Medicine) is a tertiary A-level psychiatric hospital. It is a teaching hospital of Zhejiang University and Anhui Medical University, with 1,100 beds. Among them, the Pediatric and Adolescent Psychiatry Department is the only ward in Zhejiang Province with a child psychiatric inpatient department, which has 9 doctors and 15 nurses. The service scope covers the entire Zhejiang and extends to Anhui, Jiangsu, Jiangxi, and other provinces (with a total adolescent population of over 10 million). The number of outpatient visits is over 30000 each year, of which adolescent depression patients account for 20–25%.

It was found in outpatient clinics that compared with male, female adolescent depression patients who went to the clinic for the first time were more likely to have suicidal ideas and self-harm and suicidal behaviors. According to related literature, testosterone level is closely related to impulsive behavior; therefore, this study will investigate the association between suicidal ideation and testosterone level in such patient population.

### 2.3. Measures

The primary outcome was the incidence of suicidal ideation, which was based on the Beck scale for suicide ideation (BSS) [29] and the non-suicidal self-injury behavior rating questionnaire [30]. A “General Situation Questionnaire” was developed to assess the occurrence of suicidal ideation, NSSI, and suicide attempts within a week.

This study used the “General Situation Questionnaire” to investigate the general information and self-harm and suicide of the research objects. Items include age, diagnosis, whether it is an only child, whether the parents are divorced, family history of mental disorders, and menstrual cycle.

The revised version of the Symptom Self-Rating Scale (Symptom Checklist 90, SCL-90) [31] was used to assess the clinical symptoms of patients. The scale includes 10 factors: somatization, obsessive-compulsive symptoms, interpersonal sensitivity, depression, anxiety, hostility, terror, paranoia, psychosis, and others (factors that reflect sleep and diet). A 5-point scale of 1 to 5 was used. If the total score exceeded 160 points or any factor score exceeded 2, the individual was likely to have mental health problems.

The level of testosterone was determined by the blood sample. On days 3 -5 of the menstrual cycle (if the patient has not yet had a menarche, it is not necessary to follow this time), 5 ml of venous blood was collected from the patient early in the morning (around 6:00 am) and testosterone levels were assessed using SIEMENS (ADVIA Centaru XP). The test kit (direct chemiluminescence method) measures the serum level of testosterone (sensitivity range: 0.35–52.1 nmol/L). The level of testosterone was adjusted by age, and the normal range is 0.5–2.6 nmol/L.

### 2.4. Study Participants

This study collected the first untreated adolescent female patients with depression who were hospitalized in the Seventh People's Hospital of Hangzhou from January 2018 to December 2019. Enrollment criteria: (1) female; (2) between the ages of 10 and 16 years; (3) after admission, a senior attending physician and an associate chief physician performed regular psychiatric examination, in line with ICD-10 diagnostic criteria for depression [32]; and (4) the initial depression occurred without antipsychotic medication. Exclusion criteria: (1) suffered from polycystic ovary syndrome, abnormal thyroid function, adrenal disease, pituitary tumor, or other major physical diseases; (2) neurodevelopmental disorders, autism spectrum disorder, and Asperger syndrome; (3) with impulse control disorder such as concomitant conduct disorder and hyperactivity disorder; (4) combined substance abuse of alcohol, tobacco, and drugs; (5) preexisting psychotherapy.

This study was reviewed and approved by the ethics committee of the Mental Health Center of Zhejiang University School of Medicine (IRB number: hzqy_2018_003). All subjects and their legal guardians gave informed consent to this study. Informed consent forms were obtained.

### 2.5. Statistical Analysis

Strengthening the Reporting of Observational Studies in Epidemiology (STROBE) guidelines were implemented in this study. Demographics, admission characteristics, and the SCL-90 results were described using medians and interquartile ranges for continuous variables and frequencies (%) for categorical variables. To evaluate the risk factors associated with the probability of having suicidal ideation within one week, we used multivariate logistic regression to model the suicidal ideation [33], adjusting for the continuous level of testosterone (nmol/L), age, family history of depression, and psychosis components in SCL-90. The adjusted odds ratios were reported. Furthermore, the secondary endpoints NSSI and suicide attempt were both analyzed using multivariate logistic regression, adjusting for the same covariates as listed above. The dependent variables included the self-reported incidence of the NSSI and suicide attempt.

Prior to modeling, redundancy analyses [33] were performed using an adjusted *R*^2^ cutoff of 0.6 and covariates were reduced based on the least rank in the list of available covariates. Level of statistical significance is 5%. All tests were two-sided. 95% confidence intervals were reported along with all effect estimates. R software version 3.6.4 (https://www.r-project.org/) and above were used for all the analyses.

## 3. Results

From January 2018 through December 2019, we screened 212 adolescent females, of whom 28 (13.20%) met one or more exclusion criteria (Figure 1). There were 4 (1.88%) patients or their authorized representatives who declined to participate for different reasons. Among those, 180 (84.91%) agreed to participate and signed the inform consent forms. However, 67 (31.60%) of them could not get the sample values of testosterone, due to the limited time window for the sample collection. In total, 113 (53.30%) were included in our final analysis.

A total of 113 adolescent female patients were admitted. Of the patients in this cohort, 76.11% of patients suffered from the suicidal ideation, while the percentage of patients who had experienced NSSI behaviour and suicide attempts was 52.21% and 20.35%, respectively. The mean level of testosterone was 1.7 nmol/L (0.65), and the suicidal ideation group had higher level of testosterone, compared with the naïve patients, while the same pattern did not show up in the NSSI and suicide attempt outcomes.

In the self-reported SCL-90-R, the mean of 10 domain scores for the suicidal ideation group ranged from 2.6 to 3.6, while that of the non-suicidal ideation group was lower, ranging from 2.0 to 2.7. In total, the SCL-90 total score shared the same trend of domain score, and suicidal ideation had average 66.6 lead in the comparison (Table 1).

The odds ratios for the risk factors of having suicidal ideation were presented (Table 2 and Figure 2). The testosterone level, age, and family mental disorder history were statistically significant in the model. Patients with testosterone levels of 2.03 (nmol/L) were two times more likely to experience suicidal ideation compared to those with testosterone levels of 1.19 (nmol/L). The odds ratio was 2.40 (95% CI, 1.03, 5.58), *p*=0.04. Although the family history was statistically significant, there was only one patient in the non-suicidal ideation group. It was not conclusive. There were no statistically significant differences for all the other variables.

*Note*. Differences (point estimates) in the suicidal ideation in the linear regression analyses reflect a comparison between the 25th and the 75th percentile values for each continuous variable among all 113 patients in the cohort.

## 4. Discussion

Suicidal ideation is a strong risk factor for suicidal death, and as an early stage of suicide attempts and deaths, suicidal ideation is gradually gaining attention from scholars, and timely detection and identification of patients with suicidal attempts can effectively prevent suicidal events [34]. Currently, there are few studies on suicidal ideation in depressed adolescent patients in China. Considering that the suicide rate in China is 25% higher in females than in males [35], this study selected depressed adolescent female patients and compared the age, family history of psychiatric disorders, whether they were only children, testosterone level, and other relevant factors in depressed adolescent female patients with and without suicidal ideation. The factors associated with depression in adolescent females with suicidal ideation were analyzed in order to enhance the clinical assessment of depressed adolescent patients with suicidal ideation.

In our analysis, we found that the presence of suicidal ideation is high (76.1%, 86/113). In this group of adolescent females with depression, 52.21% (59/113) had experienced NSSI behaviour and 20.35% (23/113) had attempted suicide. The incidence rate of suicidal ideation among the middle school students was 18.21% [36]. Many studies on suicide ideation among adolescents have suggested that depressive symptoms are highly correlated with suicide [34, 35, 37]. Although adolescent males are more likely to succeed in the suicide, adolescent females suffer more from suicidal ideation, NSSI, and suicidal behavior [38, 39]. Since the cases included in this study are adolescent female patients with depression, it is not uncommon that the rates of suicidal ideation, non-suicidal self-harm behavior, and suicide attempt behavior of this study are higher than those of other studies.

A 2014 Polish study's suicide data [40] showed that suicide rates were much higher among adolescents aged 15–19 years than those aged 10–14 years, which is consistent with our results. Similarly, Carballo et al. [41] found that in the United States, among adolescent children, 53% of children aged 13–19 have suicidal ideation, while only 12% of children aged 6–12 have suicidal ideation. In summary, it is not difficult to see that in adolescence, whether there is depression or not, older children seem to be more likely to have suicidal ideas, which are closely related to the physiological and psychological changes in this special period [17, 19].

Suicidal ideation in adolescents often occurs after experiencing strong negative emotions, including anxiety, restlessness, and anger [42–45]. Different from the reaction of adults experiencing negative emotions, adolescents are more likely to have suicidal ideations or destructive behaviors related to the imbalance of their emotion regulation system (ER) ability [46]. During adolescence, high levels of testosterone directly upregulate the emotional system by affecting the orbitofrontal lobe (OFC) and prefrontal cortex (PFC), destroying its stability [47, 48]. This suggests that high testosterone hormone levels may be a risk factor for a year of suicide in adolescent females with depression.

The study limitations were also evaluated. Firstly, the sample size was not large enough to attain the statistical power for all variables, such as family mental disorder history; secondly, adolescent patients with depression may modify their diagnosis as bipolar disorder in the follow-up; thirdly, the level of testosterone in adolescents may fluctuate with the menstrual cycle and the anti-depression drug may also affect the quality of the samples in this study; finally, only self-reported assessments were collected. We did not evaluate suicide conception and the frequency and severity of suicide attempts.

In conclusion, in this single-site and prospective cohort study, we found that the high level of testosterone is a potential risk factor for suicidal ideation for adolescent females who suffer from depression, especially when they are older.

## Figures and Tables

**Figure 1:** Screening, study exclusion, and enrollment.

**Figure 2:** Forest plot of odds ratios for suicidal ideation.

**Table 1:** Baseline characteristics of enrollment across the status of suicidal ideation.

	Suicidal ideation		Overall (*N* = 113)
	No (*n* = 27)	Yes (*n* = 86)	
Age (years)	12.8 (1.28)	13.7 (1.09)	13.5 (1.20)
Family mental disorder history (yes)	1 (3.70%)	18 (20.93%)	19 (16.81%)
Divorce (yes)	4 (14.81%)	9 (10.47%)	13 (11.50%)
Single child (yes)	14 (51.85%)	46 (53.49%)	60 (53.10%)
Testosterone (nmol/L)	1.4 (0.50)	1.7 (0.67)	1.7 (0.65)
SCL-90 total score	216 (61.86)	282.6 (73.14)	266.7 (75.91)
Number of positive items	59.0 (18.43)	72.5 (18.37)	69.3 (19.19)
Somatization	2.0 (0.76)	2.6 (0.99)	2.5 (0.97)
Obsessive compulsive	2.7 (0.78)	3.3 (0.84)	3.2 (0.86)
Interpersonal sensitivity	2.5 (0.81)	3.4 (0.95)	3.2 (0.99)
Anxiety	2.7 (0.88)	3.3 (1.02)	3.2 (1.02)
Depression	2.7 (0.90)	3.6 (0.91)	3.4 (0.99)
Horror	2.2 (0.79)	2.7 (0.97)	2.6 (0.95)
Hostile	2.5 (0.94)	3.3 (1.04)	3.1 (1.07)
Paranoid	2.3 (0.80)	3.1 (0.95)	2.9 (0.97)
Psychotic	2.0 (0.75)	2.8 (0.89)	2.7 (0.92)
Others	2.3 (0.79)	3.0 (0.86)	2.8 (0.90)

**Table 2:** The odds ratios of primary outcome: suicidal ideation.

	Reference	Comparison	OR (95% CI)	*p* value
Testosterone (nmol/L)	1.19	2.03	2.40 (1.03, 5.58)	0.04
Age (years)	13	14	1.74 (1.10, 2.74)	0.02
Somatization	1.67	3.25	2.18 (0.65, 7.30)	0.20
Horror	2	3.29	0.87 (0.32, 2.36)	0.78
Hostile	2.33	4	2.06 (0.63, 6.78)	0.23
Family mental disorder history	No	Yes	8.95 (1.00, 9.90)	0.05
Divorce	No	Yes	1.11 (0.23, 5.44)	0.89
Single child	No	Yes	1.50 (0.51, 4.40)	0.46

## Data Availability

The datasets used and/or analyzed during the current study are available from the corresponding author on reasonable request.
